# Natural killer/T-cell lymphoma-associated hemophagocytic syndrome: A case report

**DOI:** 10.3892/ol.2014.2202

**Published:** 2014-05-30

**Authors:** LIJUAN HAN, MINGZHI ZHANG, LING LI, LEI ZHANG, JINGJING WU, XIN LI, XINHUA WANG, KEN. H. YOUNG, XIAORUI FU, WANG MA, ZHENCHANG SUN, XUDONG ZHANG, YU CHANG, ZHI QIAO

**Affiliations:** 1 Department of Oncology, The First Affiliated Hospital of Zhengzhou University, Zhengzhou, Henan 450052, P.R. China; 2 Lymphoma Diagnosis and Treatment Center, Zhengzhou, Henan 450052, P.R. China; 3 Department of Hematopathology, University of Texas MD Anderson Cancer Center, Houston, TX 77230-1439, USA

**Keywords:** natural killer/T-cell lymphoma, hemophagocytic syndrome, clinical features, pegaspargase

## Abstract

Natural killer (NK)/T-cell lymphoma-associated hemophagocytic syndrome (HPS) is a rare and fatal disease with no optimal treatment. The present study reports the clinical features, diagnosis and treatment process of three patients with relapsed NK/T-cell lymphoma-associated HPS. All of the patients were classified as Ann Arbor stage IV and presented with a poor performance status. Two patients were successfully treated with a pegaspargase-containing combination regimen and one patient succumbed due to serious complications. These cases indicate that for patients with a history of lymphoma, the diagnosis of HPS should be considered when patients present with progressive high fever, pancytopenia and liver dysfunction. Early identification and effective treatments, including pegaspargase-based regimens are essential for an enhanced prognosis.

## Introduction

Natural killer (NK)/T-cell lymphoma is a heterogeneous and severe disease. It is rare in Europe and North America, however, more common in Asia and South America. NK/T-cell lymphoma is usually diagnosed in adults in their 50s (median age) and demonstrates a strong association with the Epstein-Barr virus (EBV). The nasal cavity and other midline facial structures are often primarily involved, as well as various aspects of the upper aerodigestive tract. NK/T-cell lymphoma is resistant to standard chemotherapy, including the CHOP regimen, which is the first-line therapy for B-cell lymphoma (1). The prognosis of NK/T-cell lymphoma is poor and may be worse when associated with hemophagocytic syndrome (HPS). HPS is characterized by a high fever, pancytopenia, splenomegaly, liver dysfunction, coagulopathy, hyperferritinemia and hemophagocytosis in the bone marrow (BM) or other organs, which is caused by high levels of inflammatory cytokines, including interferon-γ, interleukin (IL)-12, IL-18 and tumor necrosis factor-α (TNF-α) (2). The cytokine storm is a result of uncontrolled and ineffective immune activation and is triggered by underlying conditions, including infections, malignancies, autoimmune disorders and drugs, such as lamotrigine and etanercept. NK/T-cell lymphoma-associated HPS is uncommon, life-threatening and is associated with a poor prognosis, furthermore, there is no specific treatment regimen.

The current study presents three patients with relapsed NK/T-cell lymphoma-associated HPS. Two of the patients were successfully treated with a pegaspargase-containing combination regimen and supportive care. One patient succumbed due to gastrointestinal bleeding during disease progression. These cases indicate that the early identification of lymphoma-associated HPS and appropriate treatments are essential to improve patient prognosis. Patients provided written informed consent.

## Case report

### Patient A

A 22-year-old male was admitted to the Department of Oncology, the First Affiliated Hospital of Zhengzhou University (Zhengzhou, China) on 4th October 2012. The patient presented with a high fever, sore throat, congested nose and fatigue for one week. On review of the patient’s medical history it was revealed that three years previously the patient was diagnosed with extranodal NK/T-cell lymphoma, nasal type, via a biopsy of a nasal mass. Immunohistochemical analysis had revealed that the mass was positive for cluster of differentiation (CD) 3, CD43, CD56, TIA-1 and Granzyme B and negative for CD20. *In situ* hybridization for EBV-encoded early small RNAs (EBER) was also positive. The patient had been treated with six cycles of the CHOPE regimen, consisting of cyclophosphamide, doxorubicin, vincristine, prednisolone and etoposide, which had resulted in complete remission. One year previously, the patient presented with fever and purulent nasal discharge and positron emission tomography (PET) revealed hypermetabolic lesions involving the right nasal cavity and ethmoid sinus, which demonstrated recurrence of the NK/T-cell lymphoma. The patient subsequently received four cycles of gemcitabine, cisplatin and prednisolone, following which the patient’s symptoms improved along with the disappearance of the nasal mass. One week previously to the patients admission to our hospital, the patient developed a high fever of 40°C with lower extremity swelling, progressive nasal obstruction and jaundice all over the body. Due to deterioration of the condition, the patient was transferred to the Department of Oncology, the First Affiliated Hospital of Zhengzhou University for further diagnosis and treatment on the same day.

Physical examinations revealed severe jaundice of the skin and sclera, edema of the lower extremities, purulent secretion of the posterior pharyngeal wall, hepatosplenomegaly and abdominal distension with positive shifting dullness. A peripheral blood cell count revealed pancytopenia, in addition, the following results were obtained: White blood cell (WBC) count, 0.7×10^9^/l; absolute neutrophil count, 0.5×10^9^/l; hemoglobin (Hb), 108 g/l; and platelet (PLT) count, 24×10^9^/l. The results of the liver function assessments were identified to be elevated: Alanine aminotransferase (ALT), 382 U/l; aspartate aminotransferase (AST), 794 U/l; serum total bilirubin, 241 μmol/l; direct bilirubin (DBIL), 208.42 μmol/l; indirect bilirubin (IBIL), 32.6 μmol/l; and albumin (ALB), 22.7 g/l. The level of lactate dehydrogenase (LDH) was 2,532 U/l and the β2-microglobulin (β2-MG) level was elevated to 7.75 mg/l. The coagulation function showed a low level of fibrinogen (FIB; 0.79 g/l) and a prolonged activated partial thromboplastin duration (56.4 sec). Renal function parameters were within normal ranges and blood cultures were performed more than three times, with negative results. Computed tomography (CT) scans revealed bilateral pleural effusion, pericardial effusion, ascites and hepatosplenomegaly. The maxillofacial CT scan demonstrated nearly complete opacification of the bilateral maxillary and ethmoid sinus with nasal septum erosion, thus revealing the relapse of the lymphoma. Under plasma infusion, the patient underwent a BM aspirate and biopsy, which showed hemophagocytosis with no evidence of lymphoma. Further laboratory assessments revealed that the patient had high levels of serum ferritin (SF; 5,700ng ng/ml) and triglycerides (TG; 2.76 mmol/l). EBV was positive with a high replication rate (4.15×10^5^ U/ml), while the hepatitis B virus (HBV) replication rate was even higher (5.65×10^5^ U/ml). The diagnosis of NK/T-cell lymphoma-associated HPS was established based on the combination of a fever, splenomegaly, pancytopenia, hyperferritinemia, low levels of FIB and hemophagocytosis in the BM, according to the International Histiocyte Society HLH-2004 Diagnostic Criteria (3).

A DDGPE chemotherapy regimen was established, which consisted of cisplatin (20 mg/m^2^; days 1–4), dexamethasone (15 mg/m^2^; days 1–5), gemcitabine (800 mg/m^2^; day 1 and 8), pegaspargase (2,500 U/m^2^; day 1) and etoposide (100 mg; days 1–5). During chemotherapy, the patient received supportive care, including broad-spectrum antibiotics, bigeminy antivirus therapy (lamivudine and adefovir dipivoxil), plasma and PLT infusions, liver protectants and sufficient fluid supply for protection against tumor lysis syndrome. Granulocyte colony-stimulating factor (G-CSF) was administered for myelosuppression. Within three weeks of the initial chemotherapy cycle, the patient’s symptoms of fever, pancytopenia and impaired liver function improved significantly (Table I). The patient achieved partial remission with no hemophagocytosis in the BM following four cycles of DDGPE and achieved complete remission after six cycles. After almost 10 months of follow-up, the patient remained free of lymphoma-associated HPS, however, continued to present with chronic viral hepatitis with a marginally elevated HBV replication rate.

### Patient B

A 34-year-old female was admitted to the Department of Oncology, the First Affiliated Hospital of Zhengzhou University on 4th June 2013. The patient presented with fever, nausea and vomiting for 15 days. Analysis of the patient’s medical history revealed that the patient had presented with a congested nose and had undergone a nasal mass biopsy six months previously. Immunohistochemical analyses demonstrated the expression of CD2, CD3, CD56, TIA-1 and EBER, consistent with the immunophenotype of extranodal NK/T-cell lymphoma, nasal type. PET revealed involvement of the left cervical and submandibular lymph nodes, as well as the spleen and the left nasal cavity. The patient was treated with the CHOP regimen for one cycle and the DICE regimen, consisting of dexamethasone, ifosfamide, etoposide and oxaliplatin instead of cisplatin, for four cycles, following which the patient achieved partial remission. Fifteen days previously, the patient had a fever of 39.9°C and was admitted to the Department of Oncology, the First Affiliated Hospital of Zhengzhou University on 14th February 2011 for further treatment.

Physical examination showed that the patient had pale eyelid conjunctiva, splenomegaly and lower extremity edema without enlargement of the superficial lymph nodes. Laboratory assessments were conducted and revealed the following: WBC count, 2.1×10^9^/l; absolute neutrophil count, 0.8×10^9^/l; Hb, 77 g/l; and PLT count, 32×10^9^/l. Furthermore, liver function tests were observed to be abnormal as follows: ALT, 104 U/l; AST, 143 U/l; and ALB, 27.7 g/l. In addition, the patient exhibited high levels of LDH (885 U/l) and β2-MG (6.34 mg/l), as well as elevated levels of SF (3,900 ng/ml) and TG (2.46 mmol/l) and a low level of FIB (0.79 g/l). EBV was negative with a low replication rate (<5×10^2^ U/ml). Other parameters were within the normal limits. PET scanning revealed bilateral pleural effusion, pericardial effusion, hepatosplenomegaly and intense uptake of 18F-fluorodeoxyglucose in the left nasal cavity and cervical lymph nodes, which indicated the activity of the residual tumor. Furthermore, a BM aspirate and biopsy revealed hemophagocytosis, leading to the diagnosis of NK/T-cell lymphoma-associated HPS.

The patient was treated with pegaspargase (2,500 U/m^2^; day 1), dexamethasone (15 mg/m^2^; days 1–5), gemcitabine (800 mg/m^2^; day 1 and 8), etoposide (100 mg; days 1–5), cyclosporin (100 mg bid; days 1–14) and supportive treatment including human ALB and red blood cell infusions, liver protectants and nutrition support. Following the initial cycle of chemotherapy, the symptoms and laboratory parameters of the patient had improved. The patient received four cycles of chemotherapy and achieved partial remission. At present, the patient remains under treatment and is in a good condition.

### Patient C

A 58-year-old male was urgently transferred to the Department of Oncology, the First Affiliated Hospital of Zhengzhou University on 14th February 2011 presenting with a high fever, hepatosplenomegaly, enlargement of the right submandibular lymph nodes and weight loss. The records of the patient’s medical history revealed that the patient was diagnosed with NK/T-cell lymphoma, nasal type, via a biopsy of the nasal mass, 40 days previously when the patient initially presented with a fever and a congested nose. Immunohistochemical analysis identified the expression of CD3, CD43, CD56, TIA-1 and Granzyme B. The patient had received local radiotherapy for further treatment. During the radiotherapy, the patient presented with a high fever and pancytopenia. The patient was diagnosed with myelosuppression with severe infection and was treated with G-CSF and various different antibiotic regimens for almost two weeksat the People’s Hospital of Xingyang City (Xingyang, China). However, on 13th February 2011, the patient developed a higher fever, abdominal distension, and jaundice and was subsequently transferred to the Department of Oncology, the First Affiliated Hospital of Zhengzhou University with progressive deterioration of the general conditions.

The patient appeared to be anemic and exhibited jaundice, hepatosplenomegaly and enlargement of the right submandibular lymph nodes upon physical examination. Hematologic examination revealed the following: WBC count, 2.2×10^9^/l; Hb, 70 g/l; and PLT count, 30×10^9^/l. Furthermore, the serum chemistry showed abnormal results as follows: ALT, 642 U/l; AST, 514 U/l; ALB, 30.6 g/l; total bilirubin, 138 μmol/l; DBIL, 108.7 μmol/l; IBIL, 29.3 μmol/l; LDH, 702 μ/l; and β2-MG, 4.2 mg/l. SF levels were observed to be elevated to 11,816 ng/ml. The coagulation function showed a low level of FIB (0.48 g/l). An emergency CT scan revealed hepatosplenomegaly and ascites, and a BM aspirate identified the infiltration of hemophagocytosis. A diagnosis of NK/T-cell lymphoma complicated by HPS was determined.

The patient was treated with a CHOPL chemotherapy regimen consisting of cyclophosphamide (750 mg/m^2^, day 1), epirubicin (60 mg/m^2^; day 1 and 2), vincristine (2 mg/day; day 1), dexamethasone (15 mg/day; days 1–5), L-asparaginase (6,000 U/m^2^; days 3–9), as well as essential supportive treatment, including plasma and red blood cell infusions and liver protectants. The PLT and WBC counts declined progressively throughout the treatment. The patient’s symptoms progressed to a high fever and gastrointestinal bleeding over the subsequent days. Although supportive treatments were enhanced, the patient rapidly developed hemorrhagic shock. The patient’s parents chose to discontinue further treatment and the patient succumbed seven weeks after the initial presentation.

## Discussion

HPS is characterized by a high level of inflammatory cytokines secreted by activated T cells and aggressively proliferous macrophages. There are two recognized forms of HPS. Primary HPS usually presents in infants under two years old and is associated with genetic mutations, including PFR1, UNC13D and STX11. Secondary HPS is caused by underlying conditions, including infections, malignancies, autoimmune disorders and drugs, such as lamotrigine and etanercept, and is more prevalent in adults (4).

Lymphoma-associated HPS is a common type of secondary HPS, which is associated with malignancies. Han *et al* (5) reported 29 patients with lymphoma-associated hemophagocytic syndrome (LAHS) and found that the majority of cases (83%) were associated with T-cell or NK/T-cell lymphomas and exhibited a poorer prognosis compared with patients with B-cell lymphomas. The median survival time of the patients was 36 days (5). NK/T-cell lymphoma-associated HPS has rarely been reported in previous studies and is associated with a poor outcome and a high mortality rate. The symptoms of NK/T-cell lymphoma are variable, however, common presentations include a high fever, congested nose, purulent nasal discharge and an infiltrative soft tissue mass in the nasal or paranasal sinuses. The lesions may rapidly spread to neighboring and distant structures as the disease progresses. Morphologically, tissue specimens often demonstrate an angiocentric infiltration of lymphocytes with vascular invasion and tissue necrosis. Furthermore, the expression of CD3, CD56, TIA-1 and Granzyme B differentiates NK/T-cell lymphoma from other types of lymphoma.

Patient A was observed to have a high replication rate of EBV. EBV has been found to be associated with the development of NK/T-cell lymphoma. It has also been reported that EBV is significant in the development of LAHS, as well as EBV-associated HPS without lymphoma. EBV infects T cells, which may activate T lymphocytes to secret proinflammatory cytokines, including TNF-α, inducing macrophage activation. In EBV-infected T lymphocytes, expression of latent membrane protein-1 (LMP-1) has been reported. LMP-1 is a member of the TNF receptor family and activates nuclear factor κ-light-chain-enhancer of activated B cells (NF-κB). Activated NF-κB may facilitate EBV-infected T lymphocyte resistance to TNF-α-induced apoptosis, therefore, EBV-positive HPS is more likely to relapse with a poor prognosis (6,7). However, the exact pathogenesis of LAHS has yet to be elucidated. With regard to the laboratory findings, the three patients had typical presentations of HPS according to the HLH-2004 Diagnostic Criteria, including pancytopenia, low levels of FIB, hyperferritinemia, hypertriglyceridemia and hemophagocytosis in the BM. The patients also exhibited poor liver function with high levels of transaminase and bilirubin (Table II). Ost *et al* (8) performed autopsies of 27 children who had succumbed to HPS. A total of 81% of the patients presented with an infiltration of lymphocytes and a small quantity of histiocytes into the portal tracts of the liver, which was similar to the presentation of chronic persistent hepatitis (8). The study demonstrated that the liver is one of the most frequently involved organs in HPS, resulting in hepatocyte injury, and high levels of AST and ALT (8). The obstruction of the portal tracts in the liver by the infiltrating lymphocytes may explain the higher level of DBIL compared with IBIL in patients A and C, which resulted in the obstructive jaundice.

In the present study, the three patients presented with relapsed NK/T-cell lymphoma and had previously been treated with various chemotherapy regimens. Upon admission, the patients were identified to exhibit HPS with a poor performance status as the disease progressed. Early diagnosis and appropriate treatment are the two key factors for enhancing the poor prognosis. However, the complex clinical features and lack of specific symptoms complicates the early diagnosis of LAHS. NK/T-cell lymphoma is an intractable disease that is highly invasive and has no effective treatment. In NK/T lymphoma cells, there is a high expression of P-glycoprotein, which is produced by the multidrug resistance gene and exports doxorubicin and vincristine out of the cells, making NK/T lymphoma resistant to CHOP and CHOP-like regimens (9). The Asia Lymphoma Study Group reported that an L-asparaginase-containing regimen was highly effective for patients with NK/T-cell lymphoma who were newly diagnosed or had relapsed (10). L-asparaginase is an enzyme, which hydrolyzes serum L-asparagine, causing a lack of asparagine and growth inhibition in tumors that express low levels of asparagine synthetase. In the present study, pegaspargase was used instead of L-asparaginase in patients A and B, as the pegylated form of L-asparaginase leads to fewer side-effects and has a longer half-life. In addition, pegaspargase can be administered using a single injection, rather than through multiple doses as is the case with L-asparaginase (11).

Upon diagnosis of NK/T-cell lymphoma-associated HPS in patient A, the optimal treatment option was unclear. Chemotherapy with high-dose steroids and other immunosuppressive agents is essential for the treatment of LAHS; however, it may induce the fulminant replication of HBV and cause liver-associated mortality. By contrast, if antiviral and liver protection therapies were administered first, the progression of NK/T lymphoma cells and the high level of inflammatory cytokines may also be fatal to the patient. Lim *et al* (12) reported that patients who are HBV-positive and present with lymphomas show similar clinicopathological characteristics and treatment outcomes to those who are HBV-negative, therefore, should be treated similarly. Although several previous studies have reported the increased risk of liver-associated mortality and HBV reactivation during chemotherapy (13,14), the study indicated that the potential complications may be significantly reduced with the use of lamivudine (12). The control of progressive lymphoma, fulminant cytokine storms and high HBV replication rates are equally important. In the present study, patient A was treated with a pegaspargase-containing regimen that was accompanied by antivirus agents and additional supportive treatments; the patient achieved complete remission.

When patient C was initially diagnosed with NK/T-cell lymphoma, the patient was only treated with local radiotherapy, which may have been too weak for NK/T-cell lymphoma. Until hemophagocytosis was recognized in the BM in our department (Department of Oncology, Lymphoma Diagnosis and Treatment Center, Zhengzhou, China) on 19th February 2011, the patient had undergone long-term anti-infection treatment without continuous chemotherapy or further treatments in other local hospitals. The disease had reached its final and disseminated stage, resulting in the poor general condition of the patient. Despite efforts to control the progression of the disease, the patient succumbed due to serious complications.

Regarding the treatment and follow-up of patients A and B (patient B may achieve complete remission in the future), it remains unclear as to whether they should remain under observation, continue with treatment or undergo hematopoietic stem cell transplantation (HSCT). The syndrome is likely to relapse; therefore, further specific treatment should not be postponed. It was reported that the overall survival of patients with refractory or recurrent HPS following HSCT was 66% during a 6.5-year follow-up (15). Although HSCT has only occasionally been used in cases of lymphoma-associated HPS and its role in the treatment has yet to be elucidated, it may be taken into account as an opportunity to achieve long-term remission.

In conclusion, the present study demonstrates that in patients with a history of lymphoma, symptoms including fever, pancytopenia and liver dysfunction may indicate HPS, rather than the adverse side-effects of chemotherapy or radiotherapy. Early identification of HPS may facilitate the prompt and effective initiation of treatment. Once NK/T-cell lymphoma-associated HPS has been diagnosed in patients, the treatment of NK/T-cell lymphoma and HPS are particularly important. Although there is currently no optimal treatment regimen for this syndrome, active chemotherapy, including pegaspargase-based regimens are encouraged in order to prevent fatalities.

## Figures and Tables

**Table I:** Laboratory data during chemotherapy in patient A.

Time point	WBC (x10^9^/l)	Hb (g/l)	PLT (x10^9^/l)	ALT (U/l)	AST (U/l)	DBIL (μmol/l)	IBIL (μmol/l)	TBIL (μmol/l)
Pre chemo	0.7	108	24	382	794	208.4	32.6	241.0
Post chemo (days)								
3	0.6	92	16	231	294	311.6	48.1	359.8
6	0.5	84	33	309	346	128.1	32.6	160.7
9	0.3	89	41	266	128	38.9	46.5	85.4
13	0.2	102	5	114	21	64.1	31.2	95.3
19	7.5	96	172	40	32	41.7	13.4	55.1
29	6.6	97	336	43	41	18.9	7.9	26.8

Chemo, chemotherapy; WBC, white blood cell count; Hb, hemoglobin; PLT, platelet; ALT, alanine aminotransferase; AST, aspartate aminotransferase; DBIL, direct bilirubin; IBIL, indirect bilirubin; TBIL, total bilirubin.

**Table II:** Clinical features of the three patients at the time of diagnosis.

	Patient		
	
Parameter	A	B	C
Age/gender	22/M	34/F	58/M
Fever	Yes	Yes	Yes
Splenomegaly	Yes	Yes	Yes
WBC (x10^9^/l)	0.70	2.10	2.20
ANC (x10^9^/l)	0.50	0.80	1.20
Hb (g/l)	108	77	70
PLT (x10^9^/l)	24	32	30
ALT (U/l)	382	104	642
AST (U/l)	794	143	514
DBIL (μmol/l)	208.42	8.10	108.70
IBIL (μmol/l)	32.60	6.20	29.30
ALB (g/l)	22.70	27.70	30.60
LDH (U/l)	2,532	885	702
β2-MG (mg/l)	7.75	6.34	4.20
FIB (g/l)	0.79	0.79	0.48
TG (mmol/l)	2.76	2.46	-
SF (ng/ml)	5700	3900	11816
BM hemophagocytosis	Yes	Yes	Yes
EBV-DNA (U/ml)	4.15×10^5^	-	-
Stage	IV	IV	IV
ECOG	3	3	4
IPI	H	HI	H

M, male; F, female; WBC, white blood cell count; ANC, absolute neutrophil count; Hb, hemoglobin; PLT, platelets; ALT, alanine aminotransferase; AST, aspartate aminotransferase; DBIL, direct bilirubin; IBIL, indirect bilirubin; ALB, albumin; LDH, lactate dehydrogenase; β2-MG, β2-microglobulin; FIB, fibrinogen; TG, triglyceride; SF, serum ferritin; BM, bone marrow; EBV, Epstein Barr virus; ECOG, Eastern Cooperative Oncology Group scale; IPI, International Prognostic Index; H, high; HI, high intermediate.
